The article "Development Strategy of College Sports Information Management System Using Data Mining in Mobile Internet Environment" was retracted in 2023. Reasons: unreliable results or conclusions; concerns about the data; concerns about the peer review; concerns about the citations.

# Development Strategy of College Sports Information Management System Using Data Mining in Mobile Internet Environment

**DOI:** 10.1155/2022/3895555

**Published:** 2022-09-14

**Authors:** Yi Zhang

**Affiliations:** Changsha Normal University, Changsha, Hunan 410000, China

## Abstract

A strong basis has been set for the digitization of school management by the growth of big data and the Internet. However, there is not specialised software that can be used in schools to handle teaching materials and carry out teaching activities, particularly in school physical education. Most teachers struggle with significant information management issues in the conventional college sports management information system. Along with people's interest in physical education in colleges and universities, the study of the college sports management information system's development plan has emerged as the primary research area in the present day. The use of data mining in the development strategy of the sports management information system was therefore considered in conjunction with the actual situation of school sports information management. The experiment also introduced and provided a detailed explanation of the algorithm used in data mining. To fully explore the system strategy's development impact was the specific goal. In order to realise the management function of the sports management information system, serve the information management of each school, increase information management efficiency by 6.58%, and improve user satisfaction; data mining was introduced into the development strategy of management information system through the discovery of experimental data.

## 1. Introduction

People are paying greater attention to the information management system development strategy in colleges and universities as a result of the advantages of the Internet of Things that are continually emerging. Additionally, there is a growing need for sports information management at colleges and universities. However, the current college information management system's information management efficiency is insufficient to adequately meet users' expectations for sports information management. Analysis of the sports management system's development strategy using data mining technologies is therefore very important from a practical standpoint.

The methods used in information system development have been extensively examined. Lu examined the management of physical education teaching in its current state, emphasised the value of data mining in physical education instruction, and suggested a strategy for building a teaching management system [1]. Song discovered that the relationship matrix in the model could clearly depict the artificial intelligence relationship between accidents, which expanded the scope of the index analysis [2]. In order to create a cloud application platform model based on the quantity of computing resources, Wang evaluated the factors that led to the successful development of the sports education management system and integrated the concept of cloud computing [3]. In order to determine the main development direction of the International Olympic Movement in today's rapidly changing reality, Miakonkov and Enchenko employed a systematic analysis approach to identify key forward trends in the International Olympic Movement, revealing risks associated with the implementation of the goals set by the IOC [4]. Ikeda et al. developed a multimodal strategy board tool to improve Japan's competitiveness in goal kicks. It was a team sport for visually impaired players. The tool consisted of an image processing system that determines the position and movement of the ball, and a strategy board that provides tactical information [5]. A smart phone-based training information management system was created by Wang to make it easier for users to use so that they can obtain various kinds of training knowledge information [6]. To achieve high quality development, it is necessary to establish a team of teachers with a high level of professional and technical guidance. On the basis of analyzing the lack of depth in the current construction of college teachers, Warsono et al. proposed some strategies for improving the professional management team of college teachers [7]. The research results on sports information management system have been very rich, but in the process of research, many problems have been excavated.

Data mining is involved in various fields. 2.5D fighting games will be a challenging task due to the ambiguity of visual appearance such as character height or depth. Helma et al. created an OpenAI-gym-like game environment based on the network and proposed a learning Novel Networks [8]. Each machine learning and data mining technique is briefly described in a tutorial by Buczak and Guven [9]. The security of sensitive personal data is under jeopardy as a result of data mining technology's rising popularity and growth. Data suppliers, data collectors, data miners, and decision makers are the four different user categories that Xu et al. identified as being involved in data mining applications [10]. Chaurasia and Pal examined breast cancer data from the Wisconsin dataset of UCI Machine Learning [11] in order to create precise breast cancer prediction models using data mining techniques. Through their research, Yan and Zheng discovered that several basic signals continued to be significant predictors of cross-sectional stock returns even when data mining was taken into account [12]. In addition to study areas where analogous tools were being employed by the larger data mining and data science communities, Slater et al. described some of the tools emerging in educational data mining research and practise [13]. To continue combating the increase in malware samples, Ye et al. investigated intelligent malware detection methods [14]. Many people have done a lot of research on data mining technology, but few people realize the important role of applying data mining technology to college sports information management system.

Although there is a wealth of study on data mining and management information system development methodologies, outcomes that combine the two are extremely scarce. This paper combines the two in an effort to support information management. The goal of the research on the development of the information management system and its development plan is to boost the system's information management effectiveness and guarantee information security.

## 2. Data Mining Technology

### 2.1. Data Mining Structure

The main purpose of this paper is to use data mining to study the development strategy of sports management information system. However, without understanding the structure of data mining technology [15], it is difficult to use this technology to analyze the development strategy of management system. For this reason, the data mining structure is firstly analyzed, and the specific data is shown in Figure 1.

The data mining structure is divided into three parts: data modeling part, tool utilization part, and data query part. In the data modeling part, firstly, it needs to prepare the relevant data to prepare the data foundation for building the model. After the model is built, it needs to be evaluated and interpreted. Only when the evaluation effect of this model is relatively good can this model be used and consolidated. At the same time, it is also necessary to predefine a sports information management report so that users can query in time. In the tool utilization part, data mining tools and report query tools are mainly used. A professional mining tool can provide solutions to problems in a specific field. When it comes to algorithms, the particularity of data and requirements is fully considered and optimized. The report query tool can automatically calculate the corresponding statistical report according to the data in the management information system, and can create a report template that reflects the law between the data and the report. The sports information report can be automatically calculated in real time in the application based on the information in the current database as long as the parameters are supplied. Model library, database, and data warehouse are the three key modules that make up the data query portion. The model library is a model storage facility created for query reporting and data mining tools. In addition, this model library can make use of the data in relevant databases and data warehouses. According to the report query tool, the database acts as a kind of transfer station for information data that the data warehouse needs. The following is the general framework of data mining, and the data warehouse supports data mining tools.

### 2.2. Data Mining Strategy

Data mining has the potential to significantly lower the cost of managing information by properly locating query users, predicting their information demands, and providing user satisfaction. Without knowledge of the specific data mining strategy, the use of data mining theory is limited, and it is impossible to perform experiments on the information management system development strategy using data mining technology to its fullest potential [16]. As can be seen in Figure 2, this research undertakes a thorough analysis of data mining techniques.

Figure 2 shows the three main strategies in the data mining strategy, namely: unsupervised clustering [17], guided learning, and shopping basket analysis. Among them, guided learning includes three parts: classification, estimation, and prediction. Unsupervised clustering is a modeling framework in data mining. It can only be clustered into a specified number of classes, but it cannot explain the representative meaning of each class. The peculiarity of this strategy is that the algorithm used is simple and flexible enough to give reasonable results for most problems. Guided learning refers to a method of learning that is systematically guided by prescribed procedures. The information can be classified and estimated in detail according to the system guidance, and the user's query needs can be accurately predicted. Therefore, it can be applied in detail in the development strategy of the college sports information management system. Shopping basket analysis refers to a method for correlation analysis based on big data of user behavior. It can be based on basket data of all customers over a period of time. By analyzing the technical means of data mining, it can be found the hidden correlation law, which can help college sports to manage according to the correlation of its information.

### 2.3. General Process of Data Mining

The data mining technology does not end simply by screening the management information data once, but gradually penetrates into the depths of the data through multiple data screening and review. The specific data mining process is shown in Figure 3.

Figure 3 shows the seven steps of the general process of data mining: information evaluation, information understanding, data understanding, data preparation, data modeling, data evaluation, and policy deployment. First, data mining tools perform information evaluation operations on the collected relevant information. The purpose of this is to prevent some management information that does not belong to sports from being mixed in, so that the subsequent information understanding steps will be wrong. Information understanding is to conduct a deeper analysis of the evaluated information in order to obtain relevant data for research. In the data understanding step, it is necessary to understand the relevant data collected from the information, and the purpose of this is to prevent the occurrence of data collection errors. For example, the information collected in college sports information is a girl's height and weight and what she usually likes to eat, then the data collected are gender, height, and weight. The data on what girls usually like to eat does not belong to the scope of this data collection. Until the data understanding step, the data preparation work is completed. Data preparation, data modeling, data assessment, and policy deployment all build on the previous steps. Only when the first few steps are done well, can the work flow of the latter steps be relatively smooth, which in turn promotes the deployment of the development strategy of the university information management system.

### 2.4. Working Process of Data Mining in the Management System

The development plan of a collegiate sports information management system can only be better researched by people who comprehend how data mining technology in sports management systems works [18]. In order to do this, Figure 4 of this paper's general research on the operation of data mining in the management system is shown.

The data mining analysis layer, the data processing storage layer, and the data acquisition layer are three distinct examples of data mining in the information management system shown in Figure 4. The web server serves as the primary foundation for the data mining analysis layer, which also includes tools for data mining and information analysis. The primary foundation for the data processing and storage layer is the data warehouse. This data warehouse includes a model library, knowledge base, method library, and other databases. For more convenient management of the data in the data warehouse, this layer additionally offers a warehouse management function. In the data acquisition layer, internal information systems, internal Internet of Things systems, external systems, and other systems are generally present. These systems provide solid technical support for data extraction, cleaning, processing, conversion, and synthesis. On the whole, the data that has been extracted, cleaned, processed, transformed, and synthesized is the main data source of the data warehouse in the data processing storage layer. And each database in the data processing and storage layer provides analysis targets for the tools in the data mining analysis layer.

## 3. Application of Data Mining in Management System

Autoregressive models are typical modern parametric models whose autoregressive parameters contain important information about the state of the system. In time series modeling, autoregressive models are the most mature and widely used [19]. Using the autoregressive model to extract features from the data, its autoregressive parameters and residuals can be obtained as eigenvalues. When applying data mining in college sports information management, it mainly starts from this autoregressive model.

In the autoregressive model, the first step is to use the fitting formula to perform differential fitting on the time series. And this fitting formula represents the formula that the value at any moment in the random time series can be used to fit [20]:

(1) $$\begin{array}{c} x\left(n\right)=\overset{p}{\underset{i=1}{\sum }}x\left(n-1\right)+g\left(n\right), \end{array}$$

where *x* is the autoregressive parameter of the model, *P* is the model order, and *g*(*n*) is the residual error of the model.

The autoregressive model determines its own order based on the final prediction error criterion, and the calculation formula of the final prediction error criterion is:

(2) $$\begin{array}{c} P=g^{2}\frac{n+p}{n-p}, \end{array}$$

where *n* refers to the length of the sample set. If the *P* value is too small, it means that the autoregressive model fits the time series better.

Principal component analysis is an important method in statistical analysis methods and is currently widely used in feature selection and data dimensionality reduction [21]. For this reason, it is more suitable for the development strategy of college sports information management system.

Assuming that the data set *M* includes *n* samples, each sample contains *p* dimensions, then:

(3) $$\begin{array}{c} M=\left[\begin{array}{cccc} m11 & m12 & \cdots & m1p\\ m21 & m22 & \cdots & m1p\\ \vdots & \vdots & \vdots & \vdots \\ m11 & m12 & \cdots & m1p \end{array}\right]. \end{array}$$

A new indicator *F* = [*F*_1_, ⋯, *F*_*n*_] is established, which is the *p*-th principal component of the original variable, then:

(4) $$\begin{array}{c} F_{p}=u_{pp}m_{p},\\ \underset{i=0}{\sum }{u_{pi}}^{2}=1, \end{array}$$

where *u*_*pp*_ is the weighting coefficient, the new indicators *F* are not correlated, and their variances decrease in turn.

Getting the contribution rates for each component is essential to understanding the principal component analysis algorithm. The following are the key algorithmic steps:

1. The original data set *X* is standardized and transformed, and the standardized matrix *Q* is obtained
2. The correlation coefficient matrix *P* of *Q* is solved
3. The eigenvalue *k*_*i*_ of *P* and the corresponding eigenvector *l*_*i*_ are calculated, of which *k*_*i*_ are arranged in order from small to large
4. The contribution rate *C* of eigenvalue *l*_*i*_ is calculated as

(5) $$\begin{array}{c} C=\frac{k_{i}}{\Sigma_{i=1}^{p}k_{i}}. \end{array}$$

(5) The cumulative contribution rate is calculated

(6) $$\begin{array}{c} C=\frac{\Sigma_{i=1}^{b}k_{i}}{\Sigma_{i=1}^{p}k_{i}}. \end{array}$$

(6) The principal components are calculated as

(7) $$\begin{array}{c} F_{i}=l_{i}^{T}Q. \end{array}$$

(7) The principal components of the *b* principal component analysis algorithm is determined according to the contribution value

The dynamic time rounding algorithm is a commonly used method in the field of speech recognition. And sometimes in information management, it is necessary to input voice information because of the information, but the current voice input has certain defects, and the dynamic time rounding algorithm can effectively overcome this limitation. The dynamic time rounding algorithm is based on dynamic programming and can effectively measure the similarity between two time series of different lengths.

The length of the time series is:

(8) $$\begin{array}{c} \left|X\right|=\left(x_{1},\cdots x_{a}\right),\\ \left|Y\right|=\left(y_{1},\cdots y_{b}\right). \end{array}$$

The dynamic time rounding path is set to:

(9) $$\begin{array}{c} W=\left(w_{1},\cdots w_{c}\right). \end{array}$$

The dynamic time rounding path must start from 1 and end at the end of the time series. The calculation formula is:

(10) $$\begin{array}{c} \left\{\begin{array}{c} w_{c}=\left(i,j\right),\\ w_{k+1}=\left(i^{\prime },j^{\prime }\right). \end{array}\right. \end{array}$$

Among them, the sum of the minimum point-to-base distances is the dynamic time normalized distance, and the corresponding normalized path is the optimal route at this time. The dynamic time rounding distance formula is:

(11) $$\begin{array}{c} D\left(X,Y\right)=\min\left[\overset{k}{\underset{k=1}{\sum }}D_{b}\left(w_{k}\right)\right]. \end{array}$$

A cumulative distance matrix *H* with *s* rows and *t* columns is constructed:

(12) $$\begin{array}{c} F\left(s,t\right)=F_{d}\left(s,t\right)+\min F. \end{array}$$

By Formula (12), the normalized path distance of the two time series under the optimal path can be obtained.

(13) $$\begin{array}{c} r=\left\{\begin{array}{c} 1,k=\left\|x_{i}-u_{i}\right\|,\\ 0. \end{array}\right. \end{array}$$

When all samples are divided, the new center of each cluster is calculated. According to the new cluster center, the above process is repeated to divide the sample until the cluster center is stable, and its objective function is:

(14) $$\begin{array}{c} J=\overset{m}{\underset{i=1}{\sum }}\overset{K}{\underset{K=1}{\sum }}r{\left\|x_{i}-u_{k}\right\|}^{2}. \end{array}$$

The cluster center points are updated:

(15) $$\begin{array}{c} u_{k}=\underset{uk}{\min}J\left(k\right). \end{array}$$

Differentiating *u*_*k*_, the expression for *u*_*k*_ can be obtained:

(16) $$\begin{array}{c} u_{k}=\frac{\Sigma_{i}{rx}_{i}}{\Sigma_{i}r}. \end{array}$$

To understand the *k*-means algorithm in a deeper way, it is necessary to understand its calculation process. The calculation steps of the *k*-means algorithm are shown in Figure 5:

Fuzzy *C*-means clustering is a soft clustering algorithm that measures the probability of a sample data point belonging to a certain cluster according to the degree of membership. The objective function of fuzzy *C*-means clustering is:

(17) $$\begin{array}{c} J=\overset{C}{\underset{i=1}{\sum }}\underset{i=1}{\sum }u_{ij}^{m}{\left\|x_{j}-c_{i}\right\|}^{2},\\ \overset{C}{\underset{i=1}{\sum }}u_{ij}=1. \end{array}$$

In information management systems, the fuzzy *C*-means clustering method and the *k*-means algorithm are both quite helpful.

## 4. Management System Development Strategy Design

The information management system used for data mining in this paper aims to improve the management and accessibility of sports-related information. As a result, it is essential to evaluate the information management system proposed in this paper's relevant performance. In order to make the data more real and objective, this paper cites other information management systems on the Internet to compare and analyze with the efficient information management system studied in this paper. Finally, 5 users and 5 administrators are asked to use these systems according to their own information, and a questionnaire survey is conducted on their satisfaction after use. For the convenience of research, this paper names the different systems as X1, X2, X3, X4, and X5, of which system 5 is the system studied in this paper, and different users and administrators are also named according to their serial numbers. The data are shown in Table 1.

## 5. Management System Development Strategy Design Results

### 5.1. Comparison of Different Systems in terms of Management

The management system is being researched and developed to implement a more consistent management of the school's sports data. To conduct an in-depth analysis of the management effectiveness of the sports information management system under data mining, it is required to compare the management of various systems in detail in order to determine how effective each system's management is. For this reason, a comparison and analysis of the management aspects of different systems are carried out, and the specific data are shown in Figure 6.

As can be seen from Figure 6, the comparison of management aspects of different systems is mainly carried out from six aspects, such as management efficiency, stability, response time, processing speed, throughput, and management effect. In terms of management efficiency, the management efficiency of different systems was increasing from low to high. The efficiency of X1 was the lowest, only about 40%, while the management effect of X5 was the highest, up to about 90%. In terms of stability, the stability of X1 and X2 were roughly the same, and the stability was the lowest among the five systems, indicating that the stability of these two systems was far less than that of other systems. In terms of response time, the proportion of X3, X4, and X5 was the highest, much higher than several other management systems. In terms of processing speed, the proportion of X2 was the lowest among all systems, only about 57%, indicating that it took a long time to use this system. In terms of throughput, the ratios of X4 and X5 were both above 90%, which was significantly higher than that of other systems, indicating that it was not easy to cause stuttering when using these two systems. In terms of management effect, the proportion of X5 was the highest among all systems, indicating that the effect of using this system was relatively good. On the whole, the efficient information management system based on data mining technology had the best performance in management and had great practical significance. Its development strategy should focus on the research of management efficiency.

### 5.2. Comparison of Performance of Different Systems

Different systems have their own capabilities. In the detailed analysis of the information management system based on data mining, it is also necessary to study its own performance; otherwise it is very likely that the overall function has problems due to its own performance problems. In order to make the data more diverse, this paper compares and analyzes the performance of different systems, and the specific data is shown in Figure 7.

When comparing the performance of different systems, it is carried out from six aspects: operability, flexibility, convenience, fault tolerance, confidentiality, and accuracy. In terms of operability and flexibility, both X4 and X5 had the highest scores of all systems, both above 8. The scores of other systems in these two aspects were at least 1 point lower than those of the X4 and X5 systems, which mean that the operation failure was not easy to occur when the X4 and X5 systems were used. In terms of convenience, the scores of X1 and X3 were far less than those of other systems, indicating that the process was more complicated when using this system to manage information. In terms of fault tolerance, the score of X4 was about 1 point higher than that of X5, indicating that the fault tolerance of X5 needed to be improved. In terms of confidentiality, the score of X5 was significantly higher than that of other systems, indicating that when using the X5 system to manage information, it was difficult to leak management information. In terms of accuracy, the score of X3 was less than 5 points, which was the lowest among all systems, indicating that the information queried on the X3 system was prone to confusion. Although the score of X5 in fault tolerance was a little lower than that of X4, the performance of the information management system based on data mining was the best overall, and it was difficult to cause problems that greatly affect information management and query during use. The development strategy should focus on improving its fault tolerance performance.

### 5.3. Comparison of Different Systems in Terms of Cost

Each system incurs a certain cost from construction to operation and use, but the cost is not the same. For this reason, this paper compares the cost of different systems, and the specific data is shown in Figure 8.

When comparing the cost of different systems, the research is carried out from five aspects: development cost, operation cost, maintenance cost, usage cost, and management cost. In terms of development cost, X4 had the highest score among all systems, followed by X1 and X2, which had relatively high development costs, indicating that when researching the development of these three systems, the cost was relatively high. In terms of operating cost, the score of X5 was far lower than the other four management information systems, which showed that this system could save a lot of cost when running. In terms of maintenance cost, the scores of X1 and X4 were both above 7 points, which was much higher than the other three systems, indicating that the cost of maintaining these two systems was relatively high. In terms of cost of use, the score of X4 was significantly higher than that of other systems by about 2 points, indicating that a large amount of economic consumption was prone to occur when using this system. In terms of management cost, the score of X5 was less than 5 points, indicating that this system could spend less cost in managing information. On the whole, the cost consumption of the information management system based on data mining technology is relatively low in all aspects, which can save a lot of money. Therefore, its development strategy should reduce the attention of this aspect.

### 5.4. Comparison of Different Systems in Terms of Query

To develop a data mining sports information management system, it is needed to conduct research on query, but it is relatively simple to conduct strategy research only from the query function of the system itself, and no effective data can be obtained. The comparison of different systems in terms of query is analyzed, and the specific data is shown in Figure 9.

As can be seen from Figure 9, when comparing the query aspects of different systems, it is mainly compared from three aspects: query speed, query time, and query effect. In terms of query speed, the scores of X2 and X3 were the same, both below 6 points. This showed that the query speed was too slow when using these two systems to query information, which easily affected the user's experience. In terms of query time, the scores of X3 and X5 were both above 8 points, which was much higher than that of other systems, indicating that when using these two management information systems, relevant information can be queried within a period of time. In terms of query effect, the scores of X1 and X3 were relatively low among all systems, indicating that the effect of using these two systems to query information was relatively poor, and it was easy to find the problem that information cannot be queried. On the whole, the information management system based on data mining technology has better performance in query, so its development strategy should be put in a little research center.

### 5.5. Satisfaction of Different Users with Different Systems

The main purpose of researching the development strategy of information management system under data mining is to make users and administrators easy to use and improve their satisfaction. The comparison and analysis were carried out, and the specific data are shown in Figure 10.

As can be seen from Figure 10, user Y1 had the highest satisfaction with X5, which had almost reached 10 points, indicating that Y1 thought that X5 had the best use effect. User Y2 had the highest satisfaction with X4 and X5, both of which were above 8 points. User Y3's satisfaction with X1 and X3 was only about 6 points, which was the lowest score among all systems. User Y4's satisfaction with X4 was significantly higher than other management systems, indicating that Y4 thought X4 was more in line with his expectations. User Y5's satisfaction with X3 was the lowest among all systems, only about 4 points. User G1's satisfaction with X4 and X5 was the lowest among all systems, indicating that G1 thought that X4 and X5 had better management effects. User G2's satisfaction with X2 and X3 was significantly lower than other systems. Users G3, G4, and G5 had the highest satisfaction with X1, X4, and X5 among all systems, indicating that these three users thought that the management effect of X1, X4, and X5 was better. On the whole, except for the user Y4, other users were generally more satisfied with the X5, but the difference in satisfaction with the X4 was not widened. To this end, its development strategy should focus on the user's satisfaction.

## 6. Conclusion

As sports receive more and more attention from the public, more and more schools are beginning to treat sports as a professional course. However, this also means that information management system development strategies in various schools are frequently placed on the agenda. The deep level relationships between pertinent information are not taken into account in the present sports information management system development techniques, making it impossible for the management system to function as intended and completely satisfy user expectations. To provide a foundation for decision-making in physical education teaching, a thorough study of the systematic development plan has been conducted. This study compares several systems in terms of administration, performance, cost, and query, as well as the happiness of various users with various systems. It also evaluates data mining technologies and analyzes various systems collectively. The aim is to increase customer satisfaction and collect precise data on development plan. This article still has some flaws, but they will be filled in and improved upon in subsequent versions.

## Figures and Tables

**Figure 1:** Data mining structure diagram.

**Figure 2:** Data mining strategy.

**Figure 3:** General process of data mining.

**Figure 4:** Working process of data mining in the management system.

**Figure 5:** Calculation steps of *k*-means algorithm.

**Figure 6:** Comparison of different systems in terms of management.

**Figure 7:** Comparison of different systems in terms of performance.

**Figure 8:** Comparison of different systems in terms of cost.

**Figure 9:** Comparison of different systems in terms of query.

**Figure 10:** Satisfaction of different users with different systems.

**Table 1:** The specific data of the experimenter.

Personnel	Age	Weight (kg)	Height (cm)
Y1	18	55	168
Y2	21	61	171
Y3	26	45	159
Y4	34	52	163
Y5	19	59	178
G1	25	53	162
G2	21	57	167
G3	29	54	165
G4	32	55	169
G5	23	58	172

## Data Availability

The data used to support the findings of this study are available from the corresponding author upon request.
